This article has been retracted.

# Effects of Hemp Sanitary Pads on the Vaginal Microecology

**DOI:** 10.1155/2022/4435722

**Published:** 2022-10-13

**Authors:** Yange Sun, Chao Li, Yan Yan, Ailuan Lai, Xiaoxiao Peng, Xiaohong Yue, Yanling Li, Junzhuo Liu, Yan Liu

**Affiliations:** ^1^Yuetan Community Health Service Center of Fu Xing Hospital, Capital Medical University, Beijing, China; ^2^Obstetrics and Gynaecology of Fu Xing Hospital, Capital Medical University, Beijing, China; ^3^Obstetrics and Gynaecology of Daxing District People's Hospital, Beijing, China; ^4^Yayuncun Community Health Service Center, Chaoyang District, Beijing, China; ^5^Dongba Community Health Service Center, Chaoyang District, Beijing, China; ^6^Xinjiekou Community Health Service Center, Xicheng District, Beijing, China

## Abstract

**Objective:**

To evaluate the effect of hemp cotton sanitary pads on the vaginal microecology.

**Methods:**

A randomized controlled field trial was used to recruit 1002 community-based women of childbearing age. The women were randomly divided into experimental and control groups. The experimental group used hemp cotton sanitary pads, while the control group used two types of cotton sanitary randomly chosen from the top five sanitary pads in terms of market share in China. The vaginal microecology was compared between the two groups after three months.

**Results:**

According to the vaginal microecologic examination results at baseline, 1002 women were included in 3 groups: normal vaginal microecologic, vaginal microecological disorders, and suspected vaginal infections. The number of patients in three groups were 39 (3.9%), 652 (65.1%), and 311 (31%), respectively. Three months later, the vaginal microecologic status and vaginal pH value of the suspected vaginal infection group were not significantly different between the experimental group and control group. The experimental group outperformed the control group with respect to vaginal cleanliness and vaginal microecology status in the women without a vaginal infection (normal vaginal microecology or microecological disorders group). The rate of abnormal cleanliness in the experimental group was lower than the control group (31.95% [108/338] vs. 43.62% [154/353]). The incidence of suspected vaginitis in the experimental group was lower than the control group (15.29% [51/338] vs. 23.51% [83/353]).

**Conclusion:**

For women without vaginal inflammation, the use of hemp cotton sanitary pads during menstruation can help maintain the balance of the vaginal microecology to prevent reproductive tract infections.

## 1. Introduction

In normal women, there are varieties of microbes that reside in vagina and they form the normal vaginal microbiome. When combined, the vaginal microbial flora, endocrine regulation system, anatomic structure of the vagina, and local endocrine system constitute the vaginal microecosystem, which is in turn part of the entire human microecosystem. Lactobacillus, estrogen, and vaginal pH play an important role in maintaining ecological balance. Lactobacilli are usually the predominant bacteria among the normal vaginal microbial flora, sometimes living with other miscellaneous bacteria in small numbers [1]. The normal vaginal pH varies between 3.8 and 4.5. Vaginal microecologic balance is important for reducing recurrent episodes of vaginitis. Vaginal microecologic imbalance may impair the resistance to pathogenic microorganisms and increase the susceptibility to secondary infections [2]. The menstrual period is usually accompanied by a decline in the estrogen level, which alters the pH of the vagina, the vaginal microecosystem, and impairs immunity. And menstrual blood is the best medium. So, vaginitis is often occur after menstruation. The choice of appropriate sanitary pads is of high importance during the menstrual period. Hemp fibers have antibiotic and health care effects [3, 4]. Whether the use of hemp fiber-based sanitary pads in the menstrual period can improve the vaginal microecosystem and reduce infections after menstruation is a shared concern among sanitary pad manufacturers and physicians. In the present study, sanitary pads made of different materials were used, and changes in the vaginal microecosystem before and after menstruation were determined and impact of different sanitary napkins on vaginal microecology were compared.

## 2. Subjects and Methods

### 2.1. Subjects

The subjects were recruited according to the following inclusion criteria: (1) sexually active, (2) normal menstrual cycles, (3) volunteering for the present study, and (4) willingness to complete the 3-month follow-up evaluation. The exclusion criteria were a reproductive tract infection or associated symptoms in the past 1 month. All recruited patients signed an informed consent form.

### 2.2. The Research Methods

We conducted a randomized controlled field trial study by recruiting 1000 women of childbearing age from the following five community hospitals in Beijing from February to May 2021: Yuetan Community Health Service Center in Xicheng District, Xinjiekou Community Health Service Center in Xicheng District, Yayuncun Community Health Service Center in Chaoyang District, Dongba Community Health Service Center in Chaoyang District, and Beijing Daxing District People's Hospital and the Affiliated Community Health Service Center.

The patients were randomly divided into two groups (experimental and control groups). The control group was further divided into 2 subgroups. The subjects in the experimental group used hemp sanitary pads provided by Hunan Qianjin Hygienic Products Co., Ltd. (Zhuzhou, Hunan Province, China) (manufacturing filing no.: production permit no. of Hunan Medical Products Administration: 20160001), the main component of sanitary napkin is hemp cotton. As for the control group, two types of sanitary pads (both being cotton sanitary pads) were randomly chosen from the top five sanitary pads in terms of market share in China, the main component is villous pulp.

Gynecological examination and detection of vaginal discharge shall be carried out at the time of enrollment, give volunteers sanitary napkins, and inform the using of sanitary pads: (1) clean the hands before using sanitary pads, and wipe the external genitals (give the same brand of wet wipe); (2) pay attention that the hands do not touch the inner surface of the sanitary pads; (3) the replacement time is 2-3 hours/time in the daytime, and the longest is no more than 3 hours at night, according to the menstrual volume and sleep.

Secretions were detected as follows. The samples collected were submitted for evaluation within 2 h. The LTS-V800 Vaginal Discharge Analyzer (Hunan Lituo Biotechnology Co., Ltd., Hunan, China) was used for morphologic, microecologic, and chemical evaluation. The morphologic evaluation included the following: leukocytes, erythrocytes, epithelial cells, clue cells, vaginal cleanliness, and microorganisms. The chemical evaluation included the following: *β*-N-acetylglucosaminidase (NAG), neuraminidase (SNA), leukocyte esterase (LE), *β*-glucuronidase (GUS), hydrogen peroxide (H_2_O_2_), and pH value.

The test period was three menstrual period. A follow-up evaluation was performed 3-5 days after the third menstrual period ended The subjects were asked if there was any discomfort during the use of the sanitary pads. The gynecologic examination was performed to collect secretions using the same method as described above (see Figure 1). This study was approved by Medical Ethics Committee of Fuxing Hospital, Capital Medical University.

### 2.3. Observation Indices

Vaginal cleanliness, vaginal pH, and vaginal microecological examination results were used as observation indices.

The patients were divided into three groups depending on the results of the vaginal microecological evaluation (normal vaginal microecologic, vaginal microecological disorders and suspected vaginal infections).

A normal vaginal microecological was considered if all of the following criteria were met: no pathogenic microorganisms detected on morphologic evaluation, vaginal cleanliness grade I or II, 15 white blood cells/HPF, the chemical measures were normal, and the pH range was 3.8-4.5.

aginal microecological disorders was considered if all of the following criteria were met: no pathogenic microorganisms detected upon morphologic evaluation, ≤15 white blood cells/HPF, chemical evaluation of LE (+/± or H_2_O_2_+/±), and no other enzyme abnormalities.

A vaginal infection was suspected if any of the following conditions were met: pathogenic microorganisms (trichomonads, fungal hyphae or spores, and other pathogens), positive for clue cells, NAG (+), SNA (+), or GUS (+).

### 2.4. Statistical Analysis

The database was constructed using SPSS 19 software, then used for statistical analysis. Ratios were compared using a chi-square test. A *P* value < 0.05 was statistically significant.

## 3. Results

### 3.1. Baseline Information

A total of 1068 subjects were initially recruited, including 1002 patients who followed-up after menstruation and 67 patients who were lost to follow-up. The rate of lost to follow-up was 6.27%. Thus, 1002 women of childbearing age were included, with 500 subjects in the experimental group (using hemp sanitary pads) and 502 subjects in the control group. Control subgroup 1 had 252 patients, and control subgroup 2 had 250 patients. None of the patients had pruritus vulvae or an abnormal vaginal discharge. No abnormalities were noted during the gynecologic examination. The age distribution in the experimental and control groups is shown in Table 1. The two groups were matched for age; there was no significant differences in the proportion of patients in each age bracket.

### 3.2. Results of Baseline Vaginal Microecology Testing

Among the 1002 subjects, the vaginal secretion examinations showed normal vaginal cleanliness in 52.1% of the subjects (cleanliness grades I and II) and abnormal vaginal cleanliness in 47.9% of the subjects (cleanliness grades III and IV). The pH value was normal in 39.5% of the subjects (pH, 3.8-4.5) and abnormal in 60.5% of the subjects (>4.5). The patients were further divided into three subgroups based on the results of the vaginal microecology evaluation: normal microecology, microecologic disorder, and suspected vaginal infection. Subjects with a normal vaginal microecology, microecologic disorder, and suspected vaginal infection accounted for 3.9%, 65.1%, and 31%, respectively. The experimental and control groups did not differ significantly in vaginal pH values, vaginal cleanliness grades, or the results of the vaginal microecology evaluation (Table 2).

### 3.3. Results of Vaginal Secretion Examination after Intervention

Reexaminations were performed 3 months later in the experiment group which used hemp sanitary pads and the control group which used cotton sanitary pads.

#### 3.3.1. Occurrence of Vaginitis in the Past 3 Months

The incidence of vaginitis was compared. According to the results of the questionnaire survey, 29 subjects in the experimental group had vaginitis (6.3%) and 33 subjects in the control group had vaginitis (6.57%). There was no significant difference in the incidence of vaginitis between the experimental and control groups.

#### 3.3.2. Results of Vaginal Microecology Testing 3 Months Later

Upon reexaminations 3 months later, the vaginal cleanliness grade, vaginal pH value, and vaginal microecology status of the two groups are shown in Table 3. The experimental group outperformed the control group with respect to vaginal cleanliness and vaginal microecology status. A comparison between the two control subgroups did not reveal a significant difference; however, the differences were statistically significant between any other two subgroups. The experimental and control groups did not differ significantly with respect to the vaginal pH (Table 3).

#### 3.3.3. Stratification Analysis

The patients were stratified by the baseline vaginal microecology status into two groups: the group with a suspected vaginal infection and the group without a suspected vaginal infection (normal vaginal microecology or microecologic disorder). There were 691 patients who did not have a suspected vaginal infection (normal vaginal microecology or microecologic disorder). Among the 691 patients, 338 were classified into the experimental group and 353 were classified into the control group. Specifically, there were 175 subjects in control subgroup 1 and 178 subjects in control subgroup 2. There were 311 subjects with suspected vaginal infection at baseline. Among these 311 subjects, 162 were classified as the experimental group and 149 were classified as the control group.

Reexaminations were performed 3 months later. The vaginal cleanliness grade, vaginal pH, and vaginal microecology status of the patients without a vaginal infection (normal vaginal microecology or microecological imbalance) are shown in Table 4. The experimental group outperformed the control group with respect to vaginal cleanliness and vaginal microecology status. A comparison between the two control subgroups did not reveal a significant difference. The experimental and control groups did not differ significantly with respect to the vaginal pH (Table 4). The vaginal microecology status and the vaginal pH of the experimental group were not significantly different compared to the control group in patients with suspected vaginal infection.The experimental group outperformed the control group with respect to vaginal cleanliness (Table 5).

## 4. Discussion

When combined, the vaginal microbial flora, endocrine regulation system, anatomic structure of the vagina, and local endocrine system constitute the vaginal microecosystem, which is in turn part of the entire human microecosystem. Lactobacilli are usually the predominant bacteria among the normal vaginal microbial flora, sometimes living with other miscellaneous bacteria in small numbers [1]. The normal vaginal pH varies between 3.8 and 4.5. Vaginal microecologic balance is important for reducing recurrent episodes of vaginitis. Vaginal microecologic disorder may impair the resistance to pathogenic microorganisms and increase the susceptibility to secondary infections [2].

A vaginal microecologic evaluation mainly consists of morphologic and functional assessments, both of which are complementary. Such assessments offer a comprehensive evaluation of the vaginal microecologic status [5]. A vaginal microecologic evaluation has been widely used for clinical diagnosis and treatment of reproductive tract infections. This technique can also be used to identify a vaginal microecologic disorder for those who are not diagnosed clinically with reproductive tract infections. That can provide more information for clinical diagnosis and treatment [6].

Vaginal microecology is affected by many factors, and hygiene products are one of them. The safety of hygiene products has always been a concern. There are many studies on the relationship between sanitary products and reproductive tract infections, most of which focus on tampons and menstrual cups [7, 8]. There are few studies on the effect of sanitary pads on reproductive tract infection.

Hemp is one of the most fashionable plants. The huge ecological potential of the plants and the diversity of raw materials that can be delivered by the plant, makes industrial hemp interesting for agriculture, medicine, food, textiles, construction, and other industries. Hemp products also have many applications in the field of private care. It is reported that 24% of hemp products are used in private care [9].

So, compared with other sanitary pads, whether there is an impact on female reproductive tract infection? In the present study, sanitary pads made of different materials were used, and changes in the vaginal microecosystem before and after menstruation were determined. We compared the impact of different sanitary pads on vaginal microecology. The present study compared the impact of hemp and cotton sanitary pads on the vaginal microecosystem after 3 consecutive menstrual cycles. Among those with a normal vaginal microecosystem or a vaginal microecologic imbalance at baseline, the vaginal cleanliness grade and overall vaginal microecologic status were better if hemp sanitary pads were used rather than the ordinary cotton sanitary pads. In addition, there was no significant difference in the vaginal pH values between the two groups.

The improved vaginal microecologic status might be explained by the properties of hemp fibers. Two mechanisms may work simultaneously to give the antibacterial effect of hemp fibers. First, hemp fibers have strong adsorption capacity and a unique porous structure. The abundance of oxygen in the pores of the hemp fibers makes the survival of anaerobes difficult. Thus, hemp fibers inhibit bacterial growth via their unique structure. In addition, hemp fibers contain organic salts and several active phenols that kill and inhibit a variety of bacteria. Thus, hemp fibers inhibit bacterial growth via their distinct chemical composition as well [3]. One experiment showed that the inhibition rate of hemp fabric on *Staphylococcus aureus* at 1 and 4 h was 92.35% and 97.37%, respectively. The inhibition rate of hemp fabric on *Escherichia coli* was 92.27% and 96.65%, respectively [4]. Our study showed that hemp sanitary pads were indeed favorable for improving the vaginal microenvironment and maintaining a balanced vaginal microecosystem.

We also showed that among patients with a suspected vaginal infection at baseline, the vaginal microecologic status did not differ significantly after the use of hemp and ordinary cotton sanitary pads for 3 menstrual cycles. Thus, hemp sanitary pads had no therapeutic effect against vaginal infections.

A low estrogen level in the menstrual period along with the menstrual flow usually results in a higher vaginal pH value, which is conducive to the growth of pathogenic microbes. Menstrual hygiene is of high importance for preventing reproductive tract infections. Sanitary pads have become a necessity in modern society. The appropriate choice of sanitary pads is an integral part of menstrual health care. We found that hemp sanitary pads could help maintain a vaginal microecologic balance, thus reducing reproductive tract infections. Our result provides a scientific basis for preventing reproductive tract infections.

This study has at least two limitations. The total number of samples is still too small, and the follow-up time was only three months, which was relatively short. Our study may be a first step toward gathering clinical practical advice on this important issue, and in the future, we further expanded the sample size and extended the follow-up time.

## 5. Conclusion

In conclusion, in our study, for women without vaginal inflammation, the use of hemp cotton sanitary pads during menstruation can help maintain the balance of the vaginal microecology to prevent reproductive tract infections. But among patients with a suspected vaginal infection, there was no similar effect, hemp sanitary pads had no therapeutic effect against vaginal infections.

## Figures and Tables

**Figure 1:** Flow chart of research process.

**Table 1:** Age distribution of females in the experimental and control groups (*n*, %).

Age	Experimental group		Control group		Chi-square test	*P*
	Cases (*n*)	Percentage (%)	Cases (*n*)	Percentage (%)		
-30	76	15.2	77	15.33	1.943	0.379
31-39	266	53.2	286	57.0		
40-	158	31.6	139	27.7		

Total	500	100	502	100		

**Table 2:** Results of baseline vaginal secretion examinations.

Results of vaginal secretion examination		Experimental group *n* (%)	Control subgroup 1 *n* (%)	Control subgroup 2 *n* (%)	Total *n* (%)	Chi-square test	*P* value
Vaginal cleanliness	I	2 (0.4%)	3 (1.2%)	2 (0.8%)	7 (0.7%)	3.776	0.707
	II	253 (50.6%)	127 (50.4%)	135 (54%)	515 (51.4%)		
	III	104 (20.8%)	56 (22.2%)	55 (22.0%)	215 (21.5%)		
	IV	141 (28.2%)	66 (26.2%)	58 (23.2%)	264 (26.4%)		

pH value	Normal	212 (42.4%)	95 (37.7%)	89 (35.6%)	396 (39.5%)	3.692	0.158
	Abnormal	288 (57.6%)	157 (62.3%)	161 (64.4%)	606 (60.5%)		

Microecology evaluation	Normal	19 (3.8%)	11 (4.4%)	9 (3.6%)	39 (3.9%)	5.867	0.438
	disorder	319 (63.8%)	164 (65.1%)	169 (67.6%)	652 (65.1%)		
	Suspected infection	162 (32.4%)	77 (30.5%)	72 (28.8%)	311 (31%)		
Total		500 (100%)	252 (100%)	250 (100%)	1002 (100%)		

**Table 3:** Results of vaginal secretion examination in patients 3 months after use of sanitary pads (*n* = 1002).

Results of vaginal secretion examination		Experimental group	Control subgroup 1	Control subgroup 2	Total	Chi-square test	*P* value
Vaginal cleanliness	I	0 (0%)	1 (0.4%)	0 (0%)	1 (0.1%)	6.828	0.001
	II	322 (64.4%)	126 (50.0%)	135 (54%)	583 (58.2%)		
	III	86 (17.2%)	58 (23%)	64 (25.6%)	208 (20.8%)		
	IV	92 (18.4%)	67 (26.6%)	51 (20.4%)	210 (21%)		

pH value	Normal (3.8-4.5)	176 (48.5%)	90 (35.7%)	97 (39%)	363 (36.3%)	0.511	0.263
	Abnormal	324 (64.8%)	162 (64.3%)	153 (61%)	638 (63.7%)		

Microecology evaluation	Normal	12 (2.4%)	3 (1.2%)	5 (2.0%)	20 (2.0%)	6.745	0.034
	disorder	387 (77.4%)	177 (70.2%)	182 (72.8%)	746 (74.5%)		
	Suspected infection	101 (20.2%)	72 (28.6%)	63 (25.2%)	236 (23.6%)		
	Total	500	252	250	1002		

**Table 4:** Results of vaginal secretion examination in patients without a vaginal infection 3 months after sanitary pad use (*n* = 691).

Results of vaginal secretion examination		Experimental group	Control subgroup 1	Control subgroup 2	Total	Chi-square test	*P* value
Vaginal cleanliness	I	0	0	0	0	10.425	0.001
	II	230 (68%)	95 (54.3%)	104 (58.4%)	429 (62.1%)		
	III	53 (15.7%)	38 (21.7%)	44 (24.7%)	135 (19.5%)		
	IV	55 (16.3%)	42 (34.1%)	30 (16.9%)	127 (18.4%)		

pH value	Normal	114 (33.7%)	64 (36.6%)	68 (38.2%)	246 (35.6%)	1.012	0.177
	Abnormal	224 (66.3%)	111 (63.4%)	110 (61.8%)	445 (64.4%)		

Microecology evaluation	Normal	11 (3.3%)	3 (1.7%)	3 (1.7%)	17 (2.5%)	9.058	0.011
	disorder	276 (81.7%)	131 (74.9%)	133 (74.7%)	540 (78.1%)		
	Suspected infection	51 (15.1%)	41 (23.4%)	42 (23.6%)	134 (19.4%)		
	Total	338	175	178	691		

**Table 5:** Results of vaginal secretion examination in patients with a vaginal infection 3 months after sanitary pad use (*n* = 311).

Results of vaginal secretion examination		Experimental group	Control subgroup 1	Control subgroup 2	Total	Chi-square test	*P* value
Vaginal cleanliness	I	0	1 (1.3%)	0	1 (0.3%)	7.962	0.047
	II	92 (56.8%)	31 (40.3%)	31 (40.3%)	154 (49.5%)		
	III	33 (20.4%)	20 (26%)	20 (27.8%)	73 (23.5%)		
	IV	37 (22.8%)	25 (32.5%)	21 (29.2%)	83 (26.7%)		

pH value	Normal	62 (38.3%)	23 (33.8%)	30 (41.7%)	118 (37.9%)	0.016	0.497
	Abnormal	100 (61.7%)	51 (66.2%)	42 (58.3%)	193 (62.1%)		

Microecology evaluation	Normal	1 (0.6%)	0	2 (2.8%)	3 (1.0%)	1.074	0.585
	disorder	111 (68.5%)	46 (59.7%)	49 (68.1%)	206 (66.2%)		
	Suspected infection	50 (30.9%)	31 (30.4%)	21 (29.2%)	102 (32.8%)		
	Total	162	77	72	311		

## Data Availability

All data, models, and code generated or used during the study appear in the submitted article.
